# A study on interannual change features of soil salinity of cotton field with drip irrigation under mulch in Southern Xinjiang

This article has been retracted.

**DOI:** 10.1371/journal.pone.0244404

**Published:** 2020-12-30

**Authors:** Yu Zhang, Yongjun Zhu, Baolin Yao

**Affiliations:** 1 School of Geographic Sciences and Tourism, Jiaying University, Guangdong, China; 2 Paotai Soil Improvement Experimental Station, Shihezi, XinJiang, China; 3 College of Water Conservancy and Architecture Engineering, Tarim University, Alaer, XinJiang, China; University College London, UNITED KINGDOM

## Abstract

The drip irrigation under mulch has become one of significant supporting technologies for cotton industry development in Xinjiang, and has shown the good economic and ecological benefits. With the rapid development of society and economy in Southern Xinjiang, the conventional mode of large-quota winter and spring irrigation, salt leaching and alkali decreasing is difficult to support sustainable development of land and water resources in Southern Xinjiang. This study tries to adjust soil moisture and salt content regulation mode of massive water salt leaching and drip irrigation under mulch in the non-growing period of cotton field in Southern Xinjiang, explores interannual soil salinity change features of drip irrigation cotton field without winter and spring irrigation, and provides experimental basis for drip irrigation technology under mulch which can reduce and exempt cotton irrigation in winter and spring. According to ET0, the dual-factor complete combination experiment involving 3 irrigating water quotas (I1, I2, I3) and 2 irrigation times (T12, T16) was designed, and 6 treatments were involved in total(I1T12,I2T12,I3T12,I1T16,I2T16 and I3T16). The investigation results of four-year (2012–2015) field positioning experiment showed that, under the condition of “germination under drip irrigation” without winter and spring irrigation, increasing irrigation quota and irrigation times could lower 0-100cm soil salinity accumulation, but the soil salinity accumulation degree was 40-100cm, and less than 0-30cm. In the seedling stage, bud stage, blossom and boll-forming stage, and boll opening stage, the average salinity of 0-100cm soil increased by 39.81%, 31.91%, 26.85% and 29.47%, respectively. Increasing irrigation quota and irrigation times could ease interannual soil salinity accumulation degree of cotton field with drip irrigation under mulch, without winter and spring irrigation. 0-100cm soil salinity before sowing was related to the irrigation quota of cotton in the growing stage of the last year. The larger the irrigation quota was, the smaller the soil salinity before sowing would be. The accumulation amount of soil salinity at the end of growing stage under different treatments was lower than that before sowing. The drip irrigation of cotton under mulch in the growing stage could effectively regulate soil salinity distribution and space-time migration process in the growing stage of cotton. Compared with the beginning of 2012, 0-100cm average soil salinity under 3 irrigation quotas (I1, I2, I3) was 33.66%, 5.60% and 1.24%, respectively. Salt accumulating rates under 12 irrigations and 16 irrigations were 20.66% and 6.33%, respectively. The soil had the risk of salinization when the “germination under drip irrigation” without winter and spring irrigation was used. Such results can provide the reference for prevention and treatment of soil moisture and salt content of cotton field with drip irrigation under mulch in the arid region.

## 1. Introduction

The technology of drip irrigation under mulch succeeded in Xinjiang in 1996, and water conservation and salt control features of drip irrigation under mulch were prompted on a large scale in Southern Xinjiang. The research of Wang Xinying [1] showed that, soil salinity presented the trend of first increasing and then decreasing with the increase in the application years of drip irrigation under mulch. As the application years of drip irrigation under mulch extends, salinity gradually migrated and accumulated to the earth’s surface from the lower soil layer, and the soil component type had no obvious influence on the accumulation of soil salinity. Kang Yuehu [2], Dou Chaoyin [3], and Fu Hengyang [4] indicated different soil salinity change features in different years of drip irrigation. 0-40cm soil salinity of the cotton root area in Xinjiang Shihezi Paotai test station maintained at a low level for 4 consecutive years (2008–2011). 1 year later, 0-100cm soil salinity decreased by 7.9%-77.4%. Through the improvement for 3–4 years, the rate of cotton emergence could reach 60%-80%. Meanwhile, it was also found that the soil environment in the root area gradually became good with the increase of plantation years and was beneficial to the crop growth. Different drip irrigation years (0, 1, 2 and 3 years) for heavy saline soil in the shallow groundwater area could lower soil salinity of cotton root area, and the soil was in the desalination process. The research of Yin Bo [5] shows that the longer the drip irrigation years, the smaller salinity accumulation on the soil surface. At 40-60cm soil layer, salinity accumulation was more. Hudan Tumaerbai [6] studied the drip irrigation cotton field for 2-11years in Southern Xinjiang and found that 0-20cm soil salinity decreased in the period from pre-sowing to the seedling stage, increased in the boll stage, and decreased in the boll opening stage. Within the range of >40-80cm soil, soil salinity increased slowly before the sowing and gradually decreased in the boll stage—boll opening stage. At the horizontal direction, salinity accumulation gradually increased from the drip head to the mulch. At the vertical direction, the soil at 0-20cm soil layer was desalinized, and salinity accumulation degree at >60-100cm soil layer was large. In the whole cotton growing stage, 0-60cm soil presented the desalination state, and 60-100cm soil presented the salification state. Li Mingsi [7] adopted the appropriate irrigation system and good quality of water for drip irrigation of 13-year cotton field, and found that, after a fast desalination process for the 1m soil layer, soil salinity showed the dynamic equilibrium of salification and desalination, and the soil salinity would not increase with the application years of drip irrigation technology. The study of Wang Zhenhua [8] found that, under the existing irrigation system, the mean value of 0-300cm salinity was in the fast desalination stage within 3 years, and in the stable desalination stage after the application of drip irrigation for 3–8 years. After the application of drip irrigation for 8–16 years, soil salinity decreased slowly with the years of drip irrigation. The longer the application of drip irrigation was, the lower the relative salt content of the field would be. Meanwhile, the decreasing range of salinity became smaller and smaller, and would be in a dynamic equilibrium state.

Due to the special geology, climate and unreasonable development of water resources, soil salinization is more serious in Southern Xinjiang. In order to ensure the emergence of cotton seedlings, the traditional model of saline, alkali and irrigation in winter and spring is formed in the process of local cotton planting.

With the popularization of submembrane drip irrigation technology and the rapid development of social economy in Southern Xinjiang, the ratio of water supply to agricultural production is gradually reduced.

In Tarim River basin of Southern Xinjiang, the ratio of agricultural water consumption decreases, and it is difficult to further explore water-saving potential in the cotton growing stage. Under such conditions, trying the technology of drip irrigation under mulch without winter and spring irrigation is a beneficial exploration. However, there is rare research about spatial and temporal distribution of soil moisture and salt content of cotton field treated by “germination under drip irrigation” and drip irrigation under mulch in Southern Xinjiang, without winter and spring irrigation for many consecutive years. This study aims to explore the influence of no winter and spring irrigation on spatial and temporal distribution of soil moisture and salt content, and on physiological ecology of cotton, and provide the fundamental research for promoting exemption of winter and spring irrigation in Southern Xinjiang.

## 2. Material and methods

### 2.1. Experiment design

The experimental site is in the water-saving irrigation test base of College of Water Resources and Architectural Engineering, Tarim University (79°23'33"-81°53'45"E, 40°20'00"-41°47'18"N), with the altitude of 1020m, average temperature of 10.8°C, precipitation of 67.2 mm and annual evaporation capacity of 2110.5mm. It is a typical extreme arid climate zone. The soil of experimental field is mainly composed of sandy loam and loamy sand. Within 0-100cm, the soil bulk density is 1.36–1.56g/cm^3^, and pH value is 7.32–7.97. The groundwater is buried between 3.03 and 3.34m, and the groundwater salinity is between 1.56 and 2.56g/L。The precipitation mainly concentrates in May-September. The 4-year average annual precipitation was 70.61mm (The single rainfall did not exceed 5mm, so it was invalid rainfall. Therefore, the rainfall was not taken into account during the growth period of crops.) from 2012–2015.

The field test was composed of 3 irrigation quotas (I1, I2, I3) and 2 irrigation times (T12, T16), involving 6 treatments in total. The irrigating water quota was determined according to the cotton growing stage ET0. ET0 is based on the temperature, wind speed, wind direction, solar short-wave radiation, dew point, relative humidity and other data measured by the integrated weather station of self-recording American Campbell Corporation installed in the test base. Penman-Monteith formula (FAO1998) was adopted for real-time computing. The average ET_0_ from 2012 to 2015 was 1043.42mm, and the accumulative value from May to August was 631.32 mm (Table 1). The area of each test plot was 5.4×30 = 162m^2^. Each treatment was isolated with the 30cm-high and 40cm-wide balks, and the mulch with the burial depth of 50cm was laid at both sides of the balks to prevent lateral moisture seepage. The test is a multi-year continuous positioning test. For the convenience of field management, the treatment location and area remained unchanged. In the experimental field, the cotton stalks in winter remained in the field. At present, field cotton in Southern Xinjiang is mainly machine-picked. After machine-picked, the cotton stalks are left in the field, and the straw is returned to the field in the next spring. Therefore, it is a conventional practice in southern Xinjiang to leave the cotton stalks in the field in winter. Before sowing in spring, the cotton stalks were removed. Winter and spring irrigation were not conducted in 2012–2015, and “germination under drip irrigation” was adopted. Drip irrigation is a pattern of cotton seedling emergence in the spring without irrigation, such as ploughing, harrowing, laying drip irrigation belt, laying plastic film and sowing. Within 48h after sowing, drip irrigation is used for irrigation with small flow rate and small quota to make cotton seedling emergence. The experiment design is shown in Table 2. This experiment adopts the model of "dripping seedlings". Under this model, before last year’s cotton harvest, drip irrigation needs to be carried out to wash salt and store soil moisture, which is called "drip irrigation in autumn" or "drip irrigation in winter". This model is currently in the experimental stage in Southern Xinjiang.

**Table 1:** Characteristic of reference crop evapotranspiration during 2012–2015.

Year	Index	Month											
		1	2	3	4	5	6	7	8	9	10	11	12
2012	ET_0_/(mm/M)	11.59	29.81	74.10	128.27	157.55	174.51	173.55	159.20	117.52	66.15	25.13	12.10
	ET_0_/(mm/D)	0.37	1.06	2.39	4.28	5.08	5.82	5.60	5.14	3.92	2.13	0.84	0.39
2013	ET_0_/(mm/M)	14.65	32.50	59.95	132.96	176.86	179.34	165.72	151.08	102.47	63.85	23.27	9.02
	ET_0_/(mm/D)	0.47	1.16	2.00	4.43	5.71	5.98	5.35	4.87	3.42	2.06	0.78	0.29
2014	ET_0_/(mm/M)	11.32	24.24	60.67	108.64	142.58	157.22	151.59	129.40	88.04	46.29	15.15	5.58
	ET_0_/(mm/D)	0.37	0.87	1.96	3.62	4.60	5.24	4.89	4.17	2.93	1.49	0.51	0.18
2015	ET_0_/(mm/M)	10.15	24.32	68.05	111.80	145.69	160.33	168.75	131.91	90.71	49.32	21.33	9.45
	ET_0_/(mm/D)	0.33	0.87	2.20	3.73	4.70	5.34	5.44	4.26	3.02	1.59	0.71	0.30
2012-2015Average value	ET_0_/(mm/M)	11.93	27.72	65.69	120.42	155.67	167.85	164.90	142.90	99.68	56.41	21.22	9.04
	ET_0_/(mm/D)	0.38	0.99	2.14	4.01	5.02	5.59	5.32	4.61	3.32	1.82	0.71	0.29

**Table 2:** Experimental design and irrigation treatment for mulching mulch drip irrigation of cotton in 2012–2015.

growth stage	seedling stage		budding stage		blossoming and boll-forming stage		boll opening stage		total	
	Irrigating water quota	Irrigation frequency	Irrigating water quota	Irrigation frequency	Irrigating water quota	Irrigation frequency	Irrigating water quota	Irrigation frequency	Irrigating water quota	Irrigation frequency
I1T12	0.20ET_0_ (38±3)	2	0.50ET_0_ (71±5)	3	0.75ET_0_ (186±10)	5	0.40ET_0_ (59±25)	2	354±39	12
I2T12	0.25ET_0_ (48±3)		0.60ET_0_ (85±7)		0.85ET_0_ (211±10)		0.55ET_0_ (79±35)		423±49	
I3T12	0.30ET_0_ (58±3)		0.75ET_0_ (106±8)		0.95ET_0_ (236±10)		0.70ET_0_ (100±45)		500±60	
I1T16	0.20ET_0_ (38±3)	3	0.50ET_0_ (71±5)	4	0.75ET_0_ (186±10)	7	0.40ET_0_ (59±25)	2	354±39	16
I2T16	0.25ET_0_ (48±3)		0.60ET_0_ (85±7)		0.85ET_0_ (211±10)		0.55ET_0_ (79±35)		423±49	
I3T16	0.30ET_0_ (58±3)		0.75ET_0_ (106±8)		0.95ET_0_ (236±10)		0.70ET_0_ (100±45)		500±60	

Note: Irrigation quota were average during 2012 to 2015. I

Cotton plantation and drip irrigation belt laying mode are “one mulch, two belts and four rows”, with wide and narrow row arrangement. The row spacing of cotton was 30cm+60cm+30cm, and plant spacing was 10cm. The single-wing labyrinth drip irrigation belt (the drip irrigation belt rated pressure is 0.1MPa, the rated flow is 1.8 L/h) was adopted as the drip irrigation belt, with the diameter of 16mm and drip head spacing of 30cm. The measured drip head flow was 1.8L/h (as shown in Fig 1). The cotton variety is the local main variety “Xinluzhong No.28”. Field cleaning and ploughing were conducted in the middle April every year. During ploughing, 180 kg/hm^2^ urea (N content 46%), 225 kg/hm^2^ ammonium dihydrogen phosphate (N content 12%, P_2_O_5_ content 61%), and 150 kg/hm^2^ potassium sulfate and magnesium (K_2_O content 21%, MgO content 5%, S content 14%) were applied. The field was leveled; the mulch was laid; hill-seeding was conducted manually. Then, water was dripped to make the seedlings emerge. In the bud stage and boll-forming stage of cotton, 450kg/hm^2^ special fertilizer for cotton (N: P_2_O_5_: K_2_O = 16:29:6) was applied with water four times. In the growing stage, insect pests (aphid and red spider) prevention and treatment, growth regulator (mepiquat chloride) spraying and other agronomic treatments were same. The irrigation water source was well water (degree of mineralization 0.31g/L). Before drip irrigation, the water was precipitated in a 30m^3^ impounding reservoir, went through the pressure regulation pump, filter and flowmeter, and then entered the buried pipelines. 75mmPE branch pipe was installed on the experimental field. 75mm×32mm×75mm tee pipe fittings were installed at each water inlet, and the ball valve and water meter (the nominal diameter is 32mm, the flow is 12m^3^/h, and the resolution ratio is 0.00001m^3^) were installed for irrigation control and water volume recording.

**Fig 1:** Field scheme of four cotton rows with one dripping pipe under mulch mulching and soil water content sampling point (Units:m).

### 2.2 Soil salinity determination method

Soil salinity determination method: soil salinity sampling of each test plot was conducted before sowing and at 7-10d in the growing stage. The soil auger was used to take soil in each plot, and there were three soil sampling positions: between mulches (1#), under narrow row drip irrigation belt (2#), and wide row (3#), as shown in Fig 2. Since in the plantation mode of “one mulch, two belts and four rows”, the cotton root system is mainly distributed between the mulches, narrow row and wide row locations, the soil salinity at 0-100cm vertical direction and within 45cm of horizontal direction at both sides with the drip irrigation belt as the center are mainly discussed in this study. The soil sampling depth is 100cm, and 10cm interval is one layer. The soil samples of corresponding soil layer at the three locations were mixed as one plot soil sample for determination. For the wet soil of each layer, about 40g soil sample was taken. After air drying and sieving with 1mm soil sieve, 20g soil was weighed and put in the 250ml triangular flask. The water and soil were added in the 100ml distilled water according to the proportion of 1:5, and vibrated for 10min on the vibrating machine. After being placed still for 15min, the leach liquor was filtered, and DDSJ-308A conductivity meter (the measuring range is 0.000μS/cm~199.9 mS/cm, **INESA Scientific Instrument Co., Ltd)** was used to determine the electric conductivity (EC) of leach liquor. After calibration of soil salinity (g/kg) determined by residue drying method, it was converted into soil salinity mass fractiong·kg^-1^ (*y* = 0.0037*x*+1.0291, *R*^2^ = 0.976, n = 115; *y* is soil salt content, g/kg; *x* is EC, *u*S/cm). The 3 repeated data were averaged to gain the processing data.

**Fig 2:** Soil salinity changes with the age of drip irrigation.

## 3. Results

### 3.1. Interannual mean soil salinity changes in cotton growing stage from 2012 to 2015

Under the conditions of “germination under drip irrigation” without winter and spring irrigation, the mean soil salinity among different soil layers at the growth period of cotton0-100cm vertical section presented the salification trend with the increase of drip irrigation years (Fig 2). Especially after exemption of winter and spring irrigation for 3 consecutive years (2012, 2013 and 2014), soil salinity increased obviously in 2015. Besides, the salification at 0-30cm soil layer was most obvious, and the increasing range of soil salinity was maximum. As the soil depth increased, salinity accumulation range decreased. As irrigation quota and irrigation times increased, the accumulation of 0-30cm soil salinity decreased. Under the mode of “germination under drip irrigation” without winter and spring irrigation, soil salinity of cotton field accumulated interannually. The salinity accumulation degree of superficial layer was higher than that of deep layer. Increasing irrigation quota and irrigation times could lower 0-100cm soil salinity accumulation, but salinity accumulation degree at 40-100cm was smaller than that at 0-30cm. 0-30cm soil salinity presented a linear increase with the drip irrigation years, and the determination coefficient R^2^ of fitting equation was greater than 0.85(If fitting according to the logarithmic relationship, the data change relationship cannot be well represented. When fitting with the logarithmic function, its R^2^ is 0.74, which is far less than the 0.85 of the linear relationship. Therefore, it is recommended to still use the linear relationship, which can better illustrate the trend of salt increase). 40-100cm soil salinity presented a logarithmic function relation with the drip irrigation years, and the determination coefficient R^2^ was greater than 0.75. The 0-30cm annual mean soil salinity increased by 23.50%, and 40-100cm annual mean soil salinity increased by 13.82%. Therefore, the interannual soil salinity increasing trend of cotton field with drip irrigation under mulch free from winter and spring irrigation further intensifies the soil salinization risk.

### 3.2 Interannual mean soil salinity changes in cotton growing stage from 2012 to 2015

In each treatment, 0-100cm mean soil salinity accumulated as drip irrigation years extended (Fig 3). In the seedling stage, mean soil salinity within 0-100cm increased by 39.81% in each treatment. It increased by 47.52% and 34.67% respectively under 12 irrigations and 16 irrigations. In the bug stage, it increased by 31.91% on the average. It increased by 34.82% and 29.00% respectively under 12 irrigations and 16 irrigations. The soil salinity increased by 44.08%, 33.61% and 18.04% respectively under irrigation quotas I1, I2 and I3. The boll-forming stage is the same as the seedling stage. The salinity decreased under I3T12. In other treatments, salinity accumulation appeared. The mean salinity increased by 26.85% in each treatment. In the boll opening stage, the mean salinity increased by 29.47% in each treatment, and rose by 34.28% and 24.66% respectively under 12 irrigations and 16 irrigations. The salinity increased by 39.13%, 25.70% and 23.58% respectively under I1, I2 and I3. Increasing irrigation times and irrigation quota can relieve interannual soil salinity accumulation degree of cotton field with drip irrigation under mulch free from winter and spring irrigation. The fitting relation met the logarithmic function. The determination coefficient of fitting equation of logarithmic function was the highest in the seedling stage and bud stage. *R*^2^ was 0.9509 and 0.9397 respectively. The determination coefficients *R*^2^ of fitting equation in the boll-forming stage and boll opening stage were 0.5045 and 0.5861, respectively.

**Fig 3:** Salinity changes on soil depth of 0-100cm with irrigation time for differents cotton growth stage in 2012–2015.

### 3.3. Analysis of soil salinity equilibrium of cotton field with drip irrigation under mulch

Cotton stalk retention pattern was adopted in winter from 2012 to 2015. In the growing stage, under the conditions of rational irrigating water quota and irrigation times as well as increasing irrigation amount and irrigation times in the boll opening stage, S1 and S2 were used to express soil salinity before sowing and in the growing stage, and soil desalination and salification within the year and between years were calculated((S1-S2)/S1×100%). The positive desalinization ratio means the soil salinity decreases and the soil is in the desalination state. The negative desalinization ratio means the soil is in the salinity accumulation process. Intra-annual and interannual soil salinity equilibriums of drip irrigation under mulch without winter and spring irrigation from 2012 to 2015 were analyzed, as shown in Table 3. Before sowing, 0-100cm soil salinity was related to the irrigation quota in the growing stage of last year. The larger the irrigation quota, the smaller the salinity content before sowing. The soil salinity cumulant in the growing stage under each treatment was smaller than that before sowing. With drip irrigation under mulch, the irrigation in the growing stage effectively regulated soil salinity distribution and space-time migration process in cotton growing stage. After exemption of winter and spring irrigation for 4 consecutive years, soil salification appeared at the end of harvest period in 2015 and before sowing in 2012. Under each treatment, 0-100cm soil salification rate was 13.50% on the average. Increasing irrigation quota and irrigation times contributed to reducing the soil salification rate. Under I1, I2 and I3 irrigation quotas, soil salification rates were 33.66%, 5.60% and 1.24% respectively. Under 12 irrigations and 16 irrigations, soil salification rates were 20.66% and 6.33% respectively.

**Table 3:** Soil salt content(g/kg) of 0-100cm for cotton drip irrigation under mulch in 2012–2015.

TIME	I1T12	I2T12	I3T12	I1T16	I2T16	I3T16
2012S2	1.49±0.20a	1.46±0.16a	1.37±0.18ab	1.45±0.13a	1.31±0.14b	1.28±0.08b
2012S1	1.80±0.21a	1.79±0.19a	1.78±0.19a	1.79±0.21a	1.79±0.21a	1.77±0.21a
2012(S2-S1)	-0.31	-0.33	-0.41	-0.34	-0.48	-0.50
Desalination (deposition)rate/%	17.09	18.24	23.17	18.87	26.92	28.02
2013S2	2.13±1.08a	1.68±0.58ab	1.74±0.35ab	1.91±0.55ab	1.44±0.16b	1.61±0.39ab
2013S1	2.01±0.30ab	1.99±0.25ab	1.82±0.30b	2.11±0.22ab	2.13±0.54a	1.89±0.31ab
2013(S2-S1)	0.12	-0.31	-0.08	-0.20	-0.68	-0.28
Desalination (deposition)rate/%	-5.94	15.79	4.45	9.47	32.14	14.81
2014S2	1.81±0.20a	1.67±0.17ab	1.65±0.14b	1.75±0.15ab	1.67±0.16ab	1.45±0.13c
2014S1	1.52±0.23ab	1.59±0.23ab	1.39±0.13b	1.51±0.28ab	1.61±0.21a	1.41±0.06b
2014(S2-S1)	-0.29	-0.09	-0.26	-0.23	-0.06	-0.04
Desalination (deposition)rate/%	15.87	5.33	15.65	13.45	3.84	2.91
2015S2	2.71±1.01a	1.98±0.50b	1.78±0.31b	2.08±0.47b	1.79±0.37b	1.82±0.29b
2015S1	2.01±0.31a	2.01±0.31a	2.01±0.31a	2.01±0.31a	2.04±0.29a	2.01±0.31a
2015(S2-S1)	0.70	-0.03	-0.23	0.07	-0.25	-0.20
Desalination (deposition)rate/%	-34.61	1.64	11.39	-3.29	12.35	9.84
2013S2-2012S1	0.34	-0.11	-0.05	0.13	-0.34	-0.17
Desalination (deposition)rate/%	-18.78	6.02	2.68	-7.00	19.21	9.42
2014S2-2012S1	-0.28	-0.20	-0.40	-0.28	-0.18	-0.37
Desalination (deposition)rate/%	15.41	11.25	22.15	15.58	9.96	20.75
2015S2-2012S1	0.92	0.19	0.00	0.29	0.01	0.04
Desalination (deposition)rate/%	-51.01	-10.90	-0.07	-16.30	-0.30	-2.40

Note: Means within the same row followed by the different small letters are significantly different at 5% level.

## 4. Discussion

In the first 3 years of no winter and spring irrigation, 0-30cm soil desalinization rate was higher than 40-100cm soil desalinization rate. Under the same irrigation times, the desalinization rate increased with the rise of irrigation quota. This research result is consistent with some domestic research results. But after 4 consecutive years, salinity accumulated, which may be due to the accumulation of salt in winter due to freezing and thawing [9]. Some research results also indicate that long-term drip irrigation of cotton root area will lead to soil salinity accumulation [10–13]. This may be because conventional drip irrigation under mulch in Southern Xinjiang is conducted in winter and spring irrigation, and no irrigation is carried out in the boll opening stage. In North Xinjiang, some cotton fields with boll opening are irrigated at the end of boll opening stage, and the snowfall in winter is large. The different irrigation modes in the cotton growing stage lead to different interannual soil salinity changes of cotton root area with drip irrigation under mulch [8].

For the sandy soils with 0-30cm mean soil salinity of 2.03g/kg before sowing, “germination under drip irrigation” without winter and spring irrigation, and “one mulch, two bents and four rows” drip irrigation under mulch were conducted. Under the reasonable irrigation quota and irrigation times in the growing stage, soil salinity at 0-100cm soil layer in the year and interannual soil salinity in the first 3 years were in the dynamic balance, and soil salinity slightly increased in the 4^th^ year. But, after exemption of winter and spring irrigation for 4 consecutive years, 0-100cm soil salinity accumulated, and salification rate decreased with the increase of irrigation quota. With drip irrigation under mulch in Southern Xinjiang, increasing irrigation amount in boll opening stage and adopting cotton stalk retention measure could reduce salinity accumulation at the upper soil layer before sowing and make soil salinity in the growing stage and interannual soil salinity maintain a low level. In a short time, soil salinization will not happen. Since large-quota winter and spring irrigation measures, long-term use of “germination under drip irrigation” without winter and spring irrigation will lead to the risk of salinization. With the rapid popularization of the "one film, three belts and six rows" machine-picked pattern with ultra-wide film (2.05m), the surface film covering area of ultra-wide film is larger than narrow film, which changes the crop water demand and irrigation system during the growth period of cotton, so the change of soil salinity under machine-picked pattern needs to be further studied.

## 5. Conclusions

1. Based on the condition of “germination under drip irrigation” without winter and spring irrigation, the mean soil salinity of different soil layers at 0-100cm vertical section presents the salification trend with the rise of irrigation years. Increasing irrigation quota and irrigation times can lower 0-100cm soil salinity accumulation, but the soil salinity accumulation degree is 40-100cm, and less than 0-30cm.
2. The 0-100cm mean salinity increased by 39.81%, 31.91%, 26.85% and 29.47% respectively in the seedling stage, bud stage, boll-forming stage and boll opening stage. Increasing irrigation quota and irrigation times can ease interannual soil salinity accumulation degree of cotton field with drip irrigation under mulch, without winter and spring irrigation.
3. Before sowing, 0-100cm soil salinity is related to the irrigation quota in the growing stage of last year. The larger the irrigation quota, the smaller the salinity content before sowing. The soil salinity cumulant in the growing stage under each treatment is smaller than that before sowing. With drip irrigation under mulch, the irrigation in the growing stage can effectively regulate soil salinity distribution and space-time migration process in cotton growing stage. Compared with the beginning of 2012, 0-100cm average soil salinity under 3 irrigation quotas (I1, I2, I3) was 33.66%, 5.60% and 1.24%, respectively. Salt accumulating rates under 12 irrigations and 16 irrigations were 20.66% and 6.33%, respectively. The soil has the risk of salinization when the “germination under drip irrigation” without winter and spring irrigation is used.

## Supporting information

S1 Data (XLSX)
